# Cyclophilin A inhibits A549 cell oxidative stress and apoptosis by modulating the PI3K/Akt/mTOR signaling pathway

**DOI:** 10.1042/BSR20203219

**Published:** 2021-01-29

**Authors:** Zhenling Ma, Wenwen Zhang, Yaru Wu, Menghao Zhang, Lei Wang, Yihan Wang, Yi Wang, Wei Liu

**Affiliations:** 1 College of Life Sciences, Henan Agricultural University, Zhengzhou 450002, China; 2 College of Resources and Environment, Henan Agricultural University, Zhengzhou 450002, China

**Keywords:** apoptosis, Cyclophilin A, oxidative stress, reactive oxygen species

## Abstract

The excessive and inappropriate production of reactive oxygen species (ROS) can cause oxidative stress and is implicated in the pathogenesis of lung cancer. Cyclophilin A (CypA), a member of the immunophilin family, is secreted in response to ROS. To determine the role of CypA in oxidative stress injury, we investigated the role that CypA plays in human lung carcinoma (A549) cells. Here, we showed the protective effect of human recombinant CypA (hCypA) on hydrogen peroxide (H_2_O_2_)-induced oxidative damage in A549 cells, which play crucial roles in lung cancer. Our results demonstrated that hCypA substantially promoted cell viability, superoxide dismutase (SOD), glutathione (GSH), and GSH peroxidase (GSH-Px) activities, and attenuated ROS and malondialdehyde (MDA) production in H_2_O_2_-induced A549 cells. Compared with H_2_O_2_-induced A549 cells, Caspase-3 activity in hCypA-treated cells was significantly reduced. Using Western blotting, we showed that hCypA facilitated Bcl-2 expression and inhibited Bax, Caspase-3, Caspase-7, and PARP-1 expression. Furthermore, hCypA activates the PI3K/Akt/mTOR pathway in A549 cells in response to H_2_O_2_ stimulation. Additionally, peptidyl-prolyl isomerase activity was required for PI3K/Akt activation by CypA. The present study showed that CypA protected A549 cells from H_2_O_2_-induced oxidative injury and apoptosis by activating the PI3K/Akt/mTOR pathway. Thus, CypA might be a potential target for lung cancer therapy.

## Introduction

Chronic enhanced oxidative stress is a pathogenic feature of most chronic diseases, such as cancer and diabetes, as well as pulmonary, cardiovascular, kidney, and neurodegenerative diseases [1,2]. Oxidative stress usually arise from the excessive accumulation of reactive oxygen species (ROS), which include hydrogen peroxide (H_2_O_2_), superoxide anions, hydroxyl radicals, and singlet oxygen [3]. Elevated levels of ROS-induced oxidative stress can induce cancer cell death [4–6]. To prevent excessive intracellular ROS, cancer cells have been found to maintain a redox balance by increasing their antioxidant potential [7–9].

Cyclophilin A (CypA), a ubiquitously expressed protein belonging to the immunophilin family, has peptidyl-prolyl cis–trans isomerase (PPIase) activity [10–12]. Moreover, CypA regulates multiple cellular functions, including protein folding, cell signaling, inflammation, tumorigenesis, and antiviral immunity [13–17]. CypA has been reported to be overexpressed in cancer cells, including human non-small cell lung cancer [18]. Although the role of CypA in oxidative stress is not clear at this point, recently, increasingly more studies have indicated that CypA is secreted by cells in response to inflammatory stimuli or hypoxia/reoxygenation and could protect cardiac myocytes from oxidative stress-induced apoptosis via the Akt/Nox2 pathway [19–22]. CypA is secreted by VSMCs in response to oxidative stress and mediates extracellular signal-regulated kinase (ERK1/2) activation and VSMC growth by reactive oxygen species [23]. CypA also protects rat neonatal cardiomyocytes from oxidative stress-induced apoptosis, especially ROS generation [24–26]. These studies suggest that CypA may play an anti-apoptotic role in multiple cell types and oxidative stress.

PI3K/Akt signaling pathway has been proven to inhibit cell apoptosis and stimulate cell proliferation [27]. Several pro-apoptotic proteins, including Bcl-2, Bax, and Caspase-9, are the downstream targets of the PI3K/Akt pathway [28]. The activation of PI3K dependent Akt phosphorylate Bcl-2 agonist of cell death (BAD), which will disaggregate with Bcl-2, and then binds to anti-apoptotic protein 14-3-3. Consequently, Bcl-2 will inhibit cytochrome *c* release and promote cell survival [29]. In addition, phosphorylated Akt could inhibit the activity of Caspase-9, which suppress the cleavage of Caspase-3, the downstream apoptotic executive protein [30]. Subsequently, Caspase-3 cleaves the death substrate poly (ADP-ribose) polymerase (PARP), which further cleaves the DNA between nucleosomes and causes apoptosis [31].

In the present study, we report that CypA inhibits H_2_O_2_-induced oxidative damage and apoptosis in human lung carcinoma A549 cells. Furthermore, we demonstrate that extracellular CypA facilitates Bcl-2 expression and inhibits Bax, Caspase-3, Caspase-7, and PARP-1 expression. Finally, we show that CypA causes activation of the PI3K/Akt/mTOR pathway in A549 cells in response to H_2_O_2_ stimulation. Therefore, our present study identifies an important role for CypA in oxidative damage and apoptosis, which makes CypA a new potential target for lung cancer therapy.

## Materials and methods

### Cell culture and reagents

Human lung carcinoma A549 and CaLu-3 were grown in monolayers at 37°C under 5% CO_2_ and maintained in Dulbecco’s Modified Eagle’s Medium (Gibco) containing 100 units/ml penicillin and 100 μg/ml streptomycin sulfate supplemented with 10% fetal bovine serum (Gibco). After pretreating with different concentrations of hCypA (100–1000 ng/ml) for 2 h, cells were exposed to 200 μmol/l H_2_O_2_.

CypA (C3805), Cyclosporin A (CsA, SML1018), and LY294002 (L9908) were obtained from Sigma; anti-Bcl-2 antibody (15071), anti-Bax antibody (5023), anti-Caspase-3 antibody (9664), anti-Caspase-7 antibody (12827), anti-PARP-1 antibody (5625), anti-Akt (4691S), anti-p-Akt (4060S), anti-mTOR (2983T), and anti-p-mTOR (5536T) were obtained from Cell Signaling Technology.

### Cell viability analysis

Cell viability was measured with a CCK-8 assay. Briefly, A549 cells were seeded in 96-well plates and pretreated with human recombinant CypA (hCypA) at various concentrations (100–1000 ng/ml) and then treated with 200 μmol/l H_2_O_2_. After treatment, 10 μl CCK-8 solution (C0037; Beyotime Institute of Biotechnology, Haimen, China) was added to each well and incubated at 37°C for 4 h. Then, the optical density of each well was recorded using a microplate reader (Bio-Tek, Winooski, VT, U.S.A.) at 450 nm.

### Measurement of the content of LDH and MDA

A549 cells were seeded in 96-well plates and cultured for 24 h. Then, the cells were treated with hCypA at different concentrations ranging from 100 to 1000 ng/ml for 24 h. At the end of treatment, lactate dehydrogenase (LDH) activity and lipid peroxidation in a culture medium were determined using an LDH cytotoxicity assay kit (91963; Sigma–Aldrich, St. Louis, MO, U.S.A.) and malondialdehyde (MDA) ELISA (S0131S; Beyotime Institute of Biotechnology, Haimen, China) according to the manufacturer’s instructions.

### Detection of the ROS level

Accumulation of intracellular ROS was detected through a peroxide-sensitive fluorescent probe, DCFH-DA (S0033S; Beyotime Institute of Biotechnology, Haimen, China). A549 cells under different treatments were incubated with 10 µM of DCFH-DA for 30 min at 37°C. The DCF fluorescence distribution of the cells was detected by a fluorospectrophotometer analysis at an excitation wavelength of 488 nm and an emission wavelength of 535 nm.

### Detection of Caspase-3 activity

The activity of Caspase-3 was determined using a Caspase-3 Activity Kit (C1115; Beyotime Institute of Biotechnology, Haimen, China). A549 cells with different treatments were lysed and incubated with 2 mM Ac-DEVD-pNA at 37°C for 4 h. Samples were measured with an ELISA reader at an absorbance rate of 405 nm. The analysis procedure was detailed in the manufacturer’s protocol.

### Measurement of SOD and GSH-Px activities

The activities of superoxide dismutase (SOD) (S0109; Beyotime Institute of Biotechnology, Haimen, China), glutathione peroxidase (GSH-Px) (A005-1-1; Nanjing Jiancheng Bioengineering Institute, Nanjing, China), and GSH were determined in culture supernatants of A549 cells with ELISA Kits (A006-1-1; Nanjing Jiancheng Bioengineering Institute, Nanjing, China) according to the relevant protocol.

### Quantitative real-time PCR

Total RNA was isolated from cells using Trizol reagent (Invitrogen). cDNA was made from total RNA using M-MLV (Promega) according to the manufacturer’s instructions. Analysis of the relative gene expression levels was performed using a StepOnePlus PCR system (Applied Biosystems) and the following PCR primers: CypA (*PPIA*) forward, 5′-CAACCCCACCGTGTTCTTC-3′; CypA (*PPIA*) reverse, 5′-ACTTGCCACCAGTGCCATTA-3′; GAPDH, which served as an internal control for the PCR primers; GAPDH forward 5′-TTGTCTCCTGCGACTTCAACAG-3′; and GAPDH reverse 5′-GGTCTGGGATGGAAATTGTGAG-3′.

### Western blot analysis

The A549 cells were lysed. Then, the proteins were quantified using a BCA assay (23225, Thermo Scientific). An equal amount of protein samples was subjected to sodium dodecyl sulfate-polyacrylamide gel electrophoresis (SDS-PAGE) and electro-transferred to 0.22 μm polyvinylidene difluoride membranes (Millipore, HATF09025). The membranes were blocked with 5% BSA and incubated with primary antibodies at 4°C overnight. The membranes were then incubated with a secondary antibody (Jackson, 1:10,000) for 1 h at room temperature followed by three 10 min washes in TBST. The bands were visualized using an enhanced chemiluminescence (ECL) system. Data within a linear range were quantified using the ImageJ Launcher software (National Institutes of Health).

### Statistical analyses

Statistical analyses were performed using Prism 5 software (GraphPad Software, San Diego, CA). Statistics were calculated using Student’s *t*-test. *P*<0.05 was considered statistically significant.

## Results

### CypA improved cell viability in H_2_O_2_-stimulated A549 cells

To investigate whether CypA can be induced by H_2_O_2_ stimulation, quantitative real-time PCR analysis was done using mRNA extracted from the human lung carcinoma (A549) cell line exposed to H_2_O_2_ for the indicated periods of time. The CypA transcripts increased after 3 h incubation and kept increasing up to 24 h under H_2_O_2_-stimulated conditions (Figure 1A). Next, an immunoblotting analysis was done using the whole cell lysate from A549 exposed to H_2_O_2_ for the indicated periods of time. As shown in Figure 1B, a rapid increase in the CypA protein level was observed. To detect the cytotoxicity effect of human recombinant CypA (hCypA) on A549 cells, A549 cells were treated with hCypA at different concentrations ranging from 100 to 1000 ng/ml for 24 h. The LDH cytotoxicity assay showed that hCypA did not exhibit a cytotoxicity effect on A549 cells even at a concentration of 500 ng/ml (Figure 1C). Therefore, we selected the concentrations of 100, 200, and 500 ng/mL for the following experiments. Then, we used H_2_O_2_ to stimulate oxidative injury in A549 cells. A549 cells were pretreated with 500 ng/ml of hCypA for the indicated periods of time and then stimulated with H_2_O_2_ for 24 h. As shown in Figure 1D, compared with the control group, the cell viability in the H_2_O_2_ stimulation group was markedly reduced. However, treatment with hCypA at 1 h dramatically increased cell viability. Additionally, treatment with hCypA (100, 200, and 500 ng/ml) gave rise to a dose-dependent increase in cell viability (Figure 1E).

**Figure 1:** CypA improved cell viability in H_2_O_2_-stimulated A549 cells (**A**) Quantitative PCR analysis of *PPIA* mRNA levels in A549 cells treated with H_2_O_2_ (200 μM) for the indicated time periods. (**B**) Immunoblot analysis of CypA in A549 cells treated with H_2_O_2_ (200 μM) for the indicated time points. (**C**) LDH activity in culture medium of A549 cells treated with human recombinant CypA (hCypA) at different concentrations ranging from 100 to 1000 ng/ml for 24 h. (**D**) Cell viability of A549 cells pretreated with 500 ng/ml hCypA for he indicated time periods, and then stimulated with H_2_O_2_ (200 μM) for 24 h. (**E**) Cell viability of A549 cells pretreated with 100, 200, or 500 ng/ml hCypA for 2 h, and then treated with H_2_O_2_ (200 μM) for 24 h. Data information: The data are shown as the means ± SD (**A, C–E**: *n*=3). *P<0.05, **P<0.01, and ***P<0.001 (unpaired two-tailed Student’s *t*-test). The data are representative of at least three independent experiments.

### CypA suppressed oxidative stress in H_2_O_2_-stimulated A549 cells

The production of ROS and MDA and the activities of SOD and GSH-Px were examined as markers of oxidative stress, especially by H_2_O_2_. As shown in Figure 2A, intracellular ROS production was remarkably increased in the A549 cells exposed to H_2_O_2_. However, this increased ROS production was attenuated by hCypA in a dose-dependent manner. We also obtained similar results with other lung cancer cell type, such as CaLu-3 stimulated by H_2_O_2_ (Figure 2B). Importantly, ELISA showed that increased hCypA treatment reduced the MDA level and enhanced SOD, GSH-Px, and GSH activities compared with the H_2_O_2_ stimulation group (Figure 2C–F). Previous studies discovered that GSH was depleted by inhibition of GSH synthetase using buthionine sulfoximine (BSO) [32,33]. Whereas hCypA treatment increased GSH activities compared to the BSO stimulation group (Figure 2G). Collectively, CypA inhibited oxidative stress in H_2_O_2_-stimulated A549 cells.

**Figure 2:** Effect of CypA on oxidative stress in H_2_O_2_-stimulated A549 cells (**A** and **B**) The ROS production of A549 (A) or CaLu-3 (B) cells pretreated with 100, 200, or 500 ng/ml hCypA for 2 h, and then treated with H_2_O_2_ (200 μM) for 24 h. (**C**) Analysis of MDA generation of A549 cells pretreated with 100, 200, or 500 ng/ml hCypA for 2 h, and then treated with H_2_O_2_ (200 μM) for 24 h. (**D**) The levels of SOD in A549 cells pretreated with 100, 200, or 500 ng/ml hCypA for 2 h, and then treated with H_2_O_2_ (200 μM) for 24 h. (**E** and** F**) Intracellular GSH-Px (E), GSH (F) activities in A549 cells pretreated with 100, 200, or 500 ng/ml hCypA for 2 h, and then treated with H_2_O_2_ (200 μM) for 24 h. (**G**) Intracellular GSH activities in A549 cells pretreated with 100, 200, or 500 ng/ml hCypA for 2 h, and then treated with BSO (50 μM) for 24 h. Data information: The data are shown as the means ± SD (A–G: *n*=3). *P<0.05 and **P<0.01 (unpaired two-tailed Student’s *t*-test). The data are representative of at least three independent experiments.

### CypA inhibited cell apoptosis in H_2_O_2_-stimulated A549 cells

We next identified the effect of CypA on Caspase-3 activity in the H_2_O_2_-stimulated A549 cells. As shown in Figure 3A, Caspase-3 activity significantly enhanced the H_2_O_2_-stimulated A549 cells compared with the control cells, while Caspase-3 activity was restored through treatment with hCypA. Furthermore, we observed similar results of Caspase-3 activity in CaLu-3 stimulated by H_2_O_2_ (Figure 3B). Subsequently, Western blot detected the expression levels of apoptosis-related genes. We observed elevated Bcl-2 levels but also a reduction in the expression of Bax, Caspase-7, and Caspase-3 due to hCypA in H_2_O_2_-stimulated A549 compared with the H_2_O_2_ stimulation group (Figure 3C–G). To further confirm that hCypA induces the activation of Caspase-3, the cleavage of PARP was also examined by Western blot. Consistently, hCypA treatment caused the concentration-dependent proteolytic cleavage of PARP-1 (Figure 3C,H). These data indicated that CypA inhibited cell apoptosis in H_2_O_2_-stimulated A549 and CaLu-3 cells.

**Figure 3:** Effect of CypA on cell apoptosis in H_2_O_2_-stimulated A549 cells (**A** and** B**) The Caspase-3 activity of A549 (A) or CaLu-3 (B) cells pretreated with 100, 200, or 500 ng/ml hCypA for 2 h, and then treated with H_2_O_2_ (200 μM) for 24 h. (**C**) Immunoblot analysis of Bax, Bcl-2, Caspase-7, Caspase-3, and PARP-1 in A549 cells pretreated with 100, 200, or 500 ng/ml hCypA for 2 h, and then treated with H_2_O_2_ (200 μM) for 24 h. (**D**–**H**) Relative quantification analysis of Bax (D), Bcl-2 (E), Caspase-7 (F), Caspase-3 (G), and PARP-1 (H). Data information: The data are shown as the means ± SD (A,B,D–H: *n*=3). *P<0.05, **P<0.01, and ***P<0.001 (unpaired two-tailed Student’s *t*-test). The data are representative of at least three independent experiments.

### CypA induced the PI3K/Akt/mTOR pathway in H_2_O_2_-stimulated A549 cells

The down-regulation of the activation of Caspase-7 and the inactivation of the Bcl-2 family members strongly suggest the involvement of the PI3K/Akt/mTOR pathway. We, therefore, tested the expression of p-PI3K, p-Akt, and p-mTOR in H_2_O_2_-stimulated A549 cells via Western blot analysis. As shown in Figure 4A, exposure to H_2_O_2_ resulted in a considerable reduction in p-PI3K, p-Akt, and p-mTOR levels. However, hCypA-pretreated A549 cells presented a dramatic increase in the protein expressions of p-PI3K, p-Akt, and p-mTOR expressions (Figure 4B–D).

**Figure 4:** Effect of CypA on the PI3K/Akt/mTOR pathway in H_2_O_2_-stimulated A549 cells (**A**) Immunoblot analysis of the indicated proteins in A549 cells pretreated with 100, 200, or 500 ng/ml hCypA for 2 h, and then treated with H_2_O_2_ (200 μM) for 24 h. (**B**–**D**) Relative quantification analysis of p-PI3K/PI3K (B), p-Akt/Akt (C), and p-mTOR/mTOR (D). Data information: The data are shown as the means ± SD (B–D: *n*=3). *P<0.05, **P<0.01, and ***P<0.001 (unpaired two-tailed Student’s *t*-test). The data are representative of at least three independent experiments.

### Inhibition of PI3K/Akt reversed the protective effects of CypA on A549 cells

Next, a PI3K/AKT-inhibitor (LY294002) was used to block activation of the PI3K/AKT signaling pathway in A549 cells. The increased cell viability caused by hCypA (500 ng/ml) was inhibited by LY294002 (Figure 5A). In addition, LY294002 treatment advanced ROS production and Caspase-3 activity compared with the hCypA-pretreated A549 cells (Figure 5B,C). Collectively, these results clearly indicated that the PI3K/Akt/mTOR pathway mediated the protective effects of hCypA on H_2_O_2_-stimulated A549 cells.

**Figure 5:** The protective effects of CypA on H_2_O_2_-stimulated A549 were reversed by LY294002 (**A**) Cell viability of A549 cells pretreated with 500 ng/ml hCypA for 2 h, and then treated with H_2_O_2_ (200 μM), in the presence or absence of LY294006 (10 μM) for 24 h. (**B**) The ROS production of A549 cells pretreated with 500 ng/ml hCypA for 2 h, and then treated with H_2_O_2_ (200 μM), in the presence or absence of LY294006 (10 μM) for 24 h. (**C**) The Caspase-3 activity of A549 cells pretreated with 500 ng/ml hCypA for 2 h, and then treated with H_2_O_2_ (200 μM), in the presence or absence of LY294006 (10 μM) for 24 h. Data information: The data are shown as the means ± SD (A–C: *n*=3); **P<0.01 and ***P<0.001 (unpaired two-tailed Student’s *t*-test). The data are representative of at least three independent experiments.

### Peptidyl-prolyl isomerase activity is required for CypA-induced PI3K/Akt/mTOR activation

CypA belongs to the immunophilin family, whose members possess peptidyl prolyl cis–trans isomerase (PPIase) activity. CsA is an immunosuppressive drug that powerfully inhibits the PPIase activity of CypA. To investigate whether PPIase activity is required for CypA-induced PI3K/Akt/mTOR activation, hCypA was incubated with CsA and then applied to A549 cells. As shown in Figure 6A, CsA inhibited the hCypA-induced proliferation of A549 cells, while the attenuated ROS production was restored by CsA (Figure 6B). Moreover, we observed that although a mutant R55A-CypA is 100-fold less active as a PPIase [34], it failed to attenuate ROS production (Figure 6C). Importantly, CsA significantly inhibited PI3K/Akt/mTOR activation by H_2_O_2_ (Figure 6D–G). Taken together, these results indicate that PPIase activity is involved in PI3K/Akt activation by CypA.

**Figure 6:** PPIase activity is required for CypA-induced PI3K/Akt activation (**A**) Cell viability of A549 cells pretreated with CsA (100 nmol/l), along with 500 ng/ml hCypA for 2 h, and then treated with H_2_O_2_ (200 μM) for 24 h. (**B**) The ROS production of A549 cells pretreated with CsA (100 nmol/l), along with 500 ng/ml hCypA for 2 h, and then treated with H_2_O_2_ (200 μM) for 24 h. (**C**) The ROS production of A549 cells transfected for 24 h with wild-type (WT)-CypA, R55A-CypA, or control vector, and then treated with H_2_O_2_ (200 μM) for 24 h. (**D**) Immunoblot analysis of the indicated proteins in A549 cells pretreated with CsA (100 nmol/l), along with 500 ng/ml hCypA for 2 h, and then treated with H_2_O_2_ (200 μM) for 24 h. (**E**–**G**) Quantification analysis of p-PI3K/PI3K (**E**), p-Akt/Akt (**F**), and p-mTOR/mTOR (**G**). Data information: The data are shown as the means ± SD (A,B,D–F: *n*=3). *P<0.05, **P<0.01, and ***P<0.001 (unpaired two-tailed Student’s *t*-test). The data are representative of at least three independent experiments.

## Discussion

Oxidative stress has been postulated to be key a determinant of cancer-related death [35–37]. CypA is overexpressed in various cancer types and is associated with tumor invasion, metastasis, and chemoresistance [18,38–42]. However, the roles of CypA in cancer and in regulating the survival and growth of cancer cells remain obscure. In our study, the mRNA and protein levels of CypA were induced by H_2_O_2_ inA549 cells, suggesting that the induction of CypA can be triggered by H_2_O_2_ stimulation and that CypA is involved in cellular oxidative stress.

Increasing evidence is demonstrating that CypA has the capacity to enhance endogenous antioxidant enzymatic activities. For instance, overexpressed CypA markedly reduces ROS produced by cyclosporin A [25]. It has also been reported that CypA can be secreted in response to ROS in vascular smooth muscle cells [20]. Thus, it appears that the antioxidant role of CypA is at least partly crucial for the cytoprotection of overexposed CypA against H_2_O_2_ treatment. In the present study, we found that CypA significantly improved cell viability of A549 cells, decreased ROS and MDA production, and enhanced SOD, GSH and GSH-Px activities, implying that CypA attenuated oxidative injury in H_2_O_2_-induced A549 cells.

It has been reported that ROS-mediated oxidative stress may lead to apoptosis mediated by the mitochondrial, death receptor, and endoplasmic reticulum pathways [43–46]. In the mitochondrial pathway, one of the first steps is increasing the permeability of the outer mitochondrial membrane, which is regulated by Bcl-2 family members [47,48]. Thereafter, cytoplasmic Caspase signaling is activated, which contributes to the execution of apoptosis [3,49]. Our results showed that CypA treatment caused an increase in Bcl-2 and a decrease in Bax, Caspase-7, Caspase-3, as well as PARP-1. These findings suggest that CypA can protect A549 cells from H_2_O_2_-induced oxidative injury and apoptosis.

In many cancers, including lung carcinoma, the PI3K/AKT/mTOR pathway is hyperactive, thus blocking apoptosis through the regulation of downstream signaling molecules, such as inhibiting the activation of Caspase-7, as well inactivating Bcl-2 family members [50,51]. Emerging evidence has demonstrated that activation of the PI3K/Akt signaling pathway protects A549 cells from oxidative stress and apoptosis [52–54]. Intriguingly, a previous study reported that extracellular CypA promotes platelet adhesion via cluster of differentiation 147 (CD147)-mediated PI3K/Akt-signaling [55]. In the present study, we demonstrated that CypA caused a dramatic activation of the PI3K/Akt/mTOR pathway in A549 cells in response to H_2_O_2_ stimulation. Moreover, the inhibition of PI3K/Akt/mTOR blocked the protective effects of CypA on H_2_O_2_-induced oxidative injury and apoptosis in A549 cells, which suggests that the cytoprotective effects of A549 are mediated by the PI3K/Akt/mTOR signaling pathway. We also found that the cytoprotection of CypA might be dependent on its PPIase activity because the CsA, which is a well-known inhibitor of PPIase activity in CypA, also aggravates ROS generation and inhibits activation of the PI3K/Akt/mTOR pathway. Consistent with our proposal, CsA has been reported to have chemotherapeutic effects in various cancer cells, including non-small cell lung cancer [56,57]. Hence, the molecular mechanism of CypA as an antioxidant should be investigated in future studies.

In conclusion, our present study demonstrate that CypA has protective effects on H_2_O_2_-induced oxidative injury and apoptosis in A549 cells. On the one hand, these protective effects may be mediated by activation of the PI3K/Akt/mTOR signaling pathway. On the other hand, the cytoprotective role of CypA seems to depend upon its PPIase activity. Hence, the PPIase activity of CypA may be a potent chemotherapeutic target for cancer therapy. Our results indicate that CypA might be a potential therapeutic strategy against solid tumors.

## Data Availability

All data included in the present study are available from the corresponding author on reasonable request.

## Abbreviations

Akt: protein kinase B
BAD: Bcl-2 agonist of cell death
Bax: Bcl2-Associated X
Bcl-2: B-cell lymphoma-2
BSO: buthionine sulfoximine
CCK-8: cell counting kit-8
CypA: Cyclophilin A
DCF: 2′,7′-dichlorofluorescein
GSH: glutathione
GSH-Px: glutathione peroxidase
H2-DCFDA: 2′,7′-dichlorodihydrofluoresceindiacetate
H_2_O_2_: hydrogen peroxide
hCypA: human recombinant CypA
LDH: lactate dehydrogenase
MDA: malondialdehyde
mTOR: mechanistic target of rapamycin kinase
PARP-1: poly (ADP-ribose) polymerase 1
PI3K: phosphoinositide 3-kinase
ROS: reactive oxygen species
SOD: superoxide dismutase
